RETRACTED

# Hypoglycemic, anti‐inflammatory, and neuroprotective potentials of crude methanolic extract from *Acacia nilotica* L. – results of an in vitro study

**DOI:** 10.1002/fsn3.4017

**Published:** 2024-02-13

**Authors:** Abdur Rauf, Muhammad Ibrahim, Taghrid S. Alomar, Najla AlMasoud, Anees Ahmed Khalil, Muneeb Khan, Ahood Khalid, Muhammad Saeed Jan, Dorota Formanowicz, Mohammed Mansour Quradha

**Affiliations:** ^1^ Department of Chemistry University of Swabi Swabi, Anbar Khyber Pakhtunkhwa Pakistan; ^2^ Department of Chemistry, College of Science Princess Nourah bint Abdulrahman University Riyadh Saudi Arabia; ^3^ University Institute of Diet and Nutritional Sciences, Faculty of Allied Health Sciences The University of Lahore Lahore Pakistan; ^4^ Department of Human Nutrition and Dietetics, Riphah College of Rehabilitation and Allied Health Sciences Riphah International University Lahore Pakistan; ^5^ Department of Pharmacy Bacha Khan University Charsadda Khyber Pakhtunkhwa Pakistan; ^6^ Chair and Department of Medical Chemistry and Laboratory Medicine Poznan University of Medical Sciences Poznan Poland; ^7^ College of Education Seiyun University Seiyun Hadhramawt Yemen; ^8^ Pharmacy Department, Medical Sciences Aljanad University for Science and Technology Taiz Yemen

**Keywords:** 5‐LOX, *Acacia nilotica*, AChE, BChE, COX‐2, α‐amylase, α‐glucosidase

## Abstract

*Acacia nilotica* L., also known as babul, belonging to the Fabaceae family and the *Acacia* genus, is typically used for ornamental purposes and also as a medicinal plant found in tropical and subtropical areas. This plant is a rich source of bioactive compounds. The current study aimed to elucidate the hypoglycemic, anti‐inflammatory, and neuroprotective potential of *A. nilotica*'s crude methanolic extract. The results of the in vitro antidiabetic assay revealed that methanolic extract of *A. nilotica* inhibited the enzyme α‐glucosidase (IC_50_: 33 μg mL^−1^) and α‐amylase (IC_50_: 17 μg mL^−1^) in a dose‐dependent manner. While in the anticholinesterase enzyme inhibitory assay, maximum inhibition was shown by the extract against acetylcholinesterase (AChE) (637.01 μg mL^−1^) and butyrylcholinesterase (BChE) (491.98 μg mL^−1^), with the highest percent inhibition of 67.54% and 71.50% at 1000 μg mL^−1^, respectively. This inhibitory potential was lower as compared to the standard drug Galantamine that exhibited 82.43 and 89.50% inhibition at the same concentration, respectively. Moreover, the methanolic extract of *A. nilotica* also significantly inhibited the activities of cyclooxygenase 2 (COX‐2) and 5‐lipoxygenase (5‐LOX) in a concentration‐dependent manner. The percent inhibitory activity of 5‐LOX and COX‐2 ranged from 42.47% to 71.53% and 43.48% to 75.22%, respectively. Furthermore, in silico, in vivo, and clinical investigations must be planned to validate the above‐stated bioactivities of *A. nilotica*.

RETRACTED

## Graphical abstract

It can be concluded from the results of our current research that *A. nilotica* possesses varied bioactivities. Herein, we evaluated the in‐vitro anti‐diabetic properties of *A. nilotica*'s crude methanolic extract. Moreover, the experimented extract significantly inhibited the activity of cholinesterase (AChE and BChE). In a nutshell, these results will provide the scientific community with baseline data in planning and executing further in‐vivo and clinical studies to investigate the use of *A. nilotica* to treat or support the treatment of diabetes, inflammation, and Alzheimer's disease.

## 1 INTRODUCTION

Inflammation is a painful and distressing immune system response to injury, manifested by symptoms of redness, swelling, and pain (Chen et al., 2018). The inflammatory response, which includes local inflammation of blood vessels, is developed and amplified through a series of chemical reactions, including the release of inflammatory agents from various immune cells and cells that have been injured (Ahmed, 2011). The pain accompanying inflammation results from endogenous substances, specifically prostaglandins, produced from arachidonic acid (AA) through the action of cyclooxygenases, i.e., cyclooxygenase 1 (COX‐1) and cyclooxygenase 2 (COX‐2) (Duarte et al., 1988; Khan et al., 2010). The overexpression of lipoxygenase (LOX) and COX converts AA to leukotriene and prostaglandins, respectively (Shah et al., 2014). These released LOX and prostaglandin products increase the sensitivity of nociceptors, causing pain and promoting vasodilation that leads to increased capillary permeability and, eventually, edema (Muoghalu et al., 2016). Therefore, COX and LOX inhibitors are favored for peripheral pain relief and inflammation reduction (Laveti et al., 2013). Nonsteroidal anti‐inflammatory drugs (NSAIDs) are widely used to alleviate inflammation (Moore et al., 2019). Even prolonged use of NSAIDs can result in gastric and renal toxicity (Magni et al., 2021), mainly due to the nonselective inhibition of COX‐1 and COX‐2 (Roedder et al., 2017). It is believed that currently used anti‐inflammatory drugs, including opiates and non‐NSAIDs, have associated toxic effects like gastric and renal ulcers and low potentiality (Coban & Degim, 2020; Phueanpinit et al., 2018). Due to these side effects, searching for new and effective pain management and anti‐inflammatory treatments is as necessary today as ever.

Alzheimer's disease (AD) is one of the most prevailing neurological disorders affecting older adults and is the primary cause of dementia (Coban & Degim, 2020). Clinically, AD is characterized by a range of symptoms, including declining memory and language abilities, cognitive impairments, and behavioral disorders such as psychosis, anxiety, and depression, all of which deteriorate over time (Syad et al., 2012). Acetylcholine (ACh) is essential in transmitting impulses through synapses (Ayaz et al., 2017; Patri, 2019). The concentration of this neurotransmitter is reduced due to the increased activity of two key enzymes, i.e., acetylcholinesterase (AChE) and butyrylcholinesterase (BChE) (Ayaz et al., 2019). Hence, inhibitors of AChE and BChE are considered one of the therapeutic choices available to restore cholinergic activity. Most currently available approved commercial drugs for AD treatment work principally by inhibiting cholinesterase activity (Ayaz et al., 2015). On the other hand, these commercial synthetic drugs available for the treatments for AD help in managing the symptoms associated with the condition temporarily and are harmful when used for a more extended period (Yiannopoulou & Papageorgiou, 2020). Hence, developing effective, safe, and easily available drugs for treating AD is needed.

RETRACTED

Diabetes mellitus (DM) is a group of metabolic disorders with various causes characterized by persistent high blood glucose serum concentration (American Diabetes Association, 2010; Hussain et al., 2019). Uncontrolled DM leads to many complications, such as diabetic retinopathy, nephropathy, and neuropathy, arising from damage to critical tissues due to microvascular changes (Sadiq et al., 2020; Tomic et al., 2022). In addition, the risk of macrovascular changes, such as peripheral vascular disease, ischemic heart disease, stroke, and reduced quality of life, increases mortality and shortens life expectancy (Aslam et al., 2018; Moreno‐Díaz et al., 2008). To reduce hyperglycemic conditions, targets for therapy include α‐amylase and α‐glucosidase (Olaokun et al., 2013). Slowing down carbohydrate digestion and reducing glucose absorption by inhibiting both α‐amylase and α‐glucosidase help curb elevated blood glucose levels (Kajaria et al., 2013). However, commercially available drugs for inhibiting α‐amylase and α‐glucosidase have associated adverse side effects, such as flatulence, diarrhea, and stomachache, reducing their appeal as treatments (Poongunran et al., 2015). The scientific community is currently focused on finding alternatives to overcome commercial drugs' low potency and harmful effects in treating hyperglycemia and diabetes. For this purpose, natural products are being investigated extensively and have been reported as safe, effective, and less harmful options to already available drugs.

RETRACTED

Traditional medicine utilizes medicinal plants with a long history in developing countries (Pan et al., 2014). They are often used as folk remedies to treat various ailments, such as neurological, inflammatory, and diabetic conditions (Oguntibeju, 2018). For centuries, herbal remedies have been used effectively in medication against various syndromes. Due to their relatively harmless effects, natural products have garnered modern scientists' attention for treating and managing various challenging diseases (Yeung et al., 2018). Plant‐derived extracts and isolates have been investigated as a safe and effective alternative to currently available synthetic compounds. Besides being a source of antioxidants, these natural constituents possess various pharmacological properties like antiviral, anticancer, anti‐inflammatory, neuroprotective, antidiabetic, and many more (Uwineza & Waśkiewicz, 2020). *Acacia nilotica* (L.) Wild, a member of the Fabaceae family, is commonly referred to as the Indian gum arabic tree, kikar, or babul, which has gained recognition as a versatile and valuable tree species. Although it is considered a nuisance weed due to its invasive nature, it has significant environmental value and holds the potential to boost the economy. *A. nilotica* has medicinal properties as per Unani, traditional Chinese medicine (TCM), and Ayurvedic texts. On the other hand, several preclinical and clinical studies support the potential functional and nutraceutical use of *A. nilotica*, owing to its diversified phytochemistry and bioactivities (Abduljawad, 2020; Saeedi et al., 2020). This plant's polyphenolic extract reportedly helps reduce induced neurotoxicity and oxidative stress conditions in an animal model (Foyzun et al., 2022). Moreover, *A. nilotica* extract restored glucose homeostasis by inhibiting JNK (c‐Jun N‐terminal kinase) and upregulation of insulin (Majeed et al., 2021). In diabetic rats, *A. nilotica*'s extracts lowered cholesterol levels and imparted renoprotective effects (Niyodusenga et al., 2019; Sirajo et al., 2022). Quercetin, kaempferol, and ellagic acid present in the extracts of *A*. *nilotica* are considered responsible for this plant's diverse biological activities (Al‐Nour et al., 2019). Given the importance of *A. nilotica*, the current study was designed to investigate the hypoglycemic, anti‐inflammatory, and neuroprotective potential of *Acacia nilotica*'s crude methanolic extract.

## 2 MATERIALS AND METHODS

### 2.1 Plant collection

The stems of *A. nilotica* were collected from Swabi, Khyber Pakhtunkhwa province (KPK), Pakistan, and were brought to the Department of Botany, University of Swabi (UoS), Khyber Pakhtunkhwa (KP), Pakistan, for authentication. Specimens were placed in the herbarium of UoS with voucher no. (UOS/Bot‐121).

RETRACTED

### 2.2 Extraction

The *A. nilotica* stems were collected thoroughly, washed with tap water, and shade‐dried for 10 days. The dried stem was ground into a fine powder (40 mesh) using a laboratory mill (Haier, HJE‐1024). Stem powder (100 g) was placed in a thimble, and methanol (70%) was used for extraction. The extract was placed in a clean flat‐bottomed flask, left to soak for 72 h with periodic stirring, and was later stored at room temperature in sterile bottles. Whatman No. 1 filter paper was used to filter the extract, which was subsequently concentrated using a rotary concentrator (Rotavapor® R‐300, BUCHI Corporation, USA) (Revathi et al., 2017).

### 2.3 Antidiabetic activity

#### 2.3.1 In vitro α‐amylase inhibition assay

Already established protocols for the evaluation of the α‐amylase inhibitory potential of *A. nilotica*'s crude methanolic extract were followed in this study (Huneif et al., 2022). Phosphate buffer was used for the preparation of the α‐amylase solution. Varied concentrations (62.5–1000 μg mL^−1^) of crude methanolic extract (30 μL) were mixed with already prepared α‐amylase solution (10 μL) and phosphate buffer (pH: 6.9; 2 mM). This experiment used acarbose (64 mg mL^−1^) as a positive control. The prepared mixtures were initially incubated at 25°C for 10 min. Afterwards, the reaction was initiated by adding starch solution (1%; 40 mL) in test samples and control‐containing tubes and was incubated again (10 min; 25°C). Later, iodine solution (75 μL) and hydrochloric acid (HCl) (20 μL; 1 M) were added to end the reaction, and absorbance (Abs) was measured at 540 nm. The below‐mentioned formula was used for calculating the percent inhibition of α‐amylase activity:

$$\%\text{inhibition}=\left[\frac{\mathrm{Abs}.\;\text{of control}-\mathrm{Abs}.\;\text{of test sample}}{\mathrm{Abs}.\;\text{of control}}\right]\times 100$$

#### 2.3.2 In vitro α‐glucosidase inhibitory assay

In this assay, *A. nilotica*'s crude methanolic extract was examined for its α‐glucosidase inhibitory potential by following the protocols adopted by Revathi et al. (2017). For this purpose, varied concentrations (62.5–1000 μg mL^−1^) of 50 μL of crude extract and acarbose were allowed to incubate (37°C; 20 min) with α‐glucosidase solution (10 μL; 1 U mL^−1^) and phosphate buffer (0.1 M; 125 μL; pH: 6.9). Afterwards, the reaction was initiated by adding substrate (1 M 4‐nitrophenyl β‐D‐glucopyranoside (pNPG); 20 μL). This mixture was allowed to incubate at 37°C for further 30 min. Later, 50 μL of sodium carbonate (Na_2_CO_3_) (0.1 N) was added to this mixture to stop the reaction. Finally, the absorbance (Abs) of the control and the test samples (containing crude methanolic extract) was calculated at 405 nm. Herein, acarbose was used as a positive control. α‐Glucosidase inhibition was deduced from the following formula:

$$\%\text{inhibition}=\left[\frac{\mathrm{Abs}.\;\text{of control}-\mathrm{Abs}.\;\text{of test sample}}{\mathrm{Abs}.\;\text{of control}}\right]\times 100$$

RETRACTED

### 2.4 In vitro anticholinesterase inhibitory activity

To assess the AChE and BChE inhibitory potentials of *A. nilotica*'s crude methanolic extract, the in vitro anticholinesterase assay followed the already reported protocols (Huneif et al., 2022). Varied concentrations (62.5–1000 μg mL^−1^) of crude extract and standard drug Galantamine were prepared and used in this assay. The IC_50_ values were calculated by creating a graph in Excel that compared the inhibition and concentration of the sample solution being tested.

### 2.5 Anti‐inflammatory activity

#### 2.5.1 Cyclooxygenase (COX‐2) assay

The COX‐2 assay was performed to assess the anti‐inflammatory potential of *A. nilotica*'s crude methanolic extract through the protocols reported by Jan et al. (2020). This assay prepared a solution containing 300 U mL^−1^ of the COX‐2 enzyme. For the activation of the enzyme, its solution (10 mL) was kept on ice for 5–10 min. Additionally, the enzyme solution was combined with a cofactor solution [(50 mL); hematin: 1 mM; glutathione: 0.9 mM; TMPD (N,N,N',N'‐tetramethyl‐p‐phenylenediamine dihydrochloride): 0.24 mM] prepared in Tris–HCl buffer (0.1 M, pH: 8). Afterwards, the extract (62.5–1000 mg mL^−1^) and the enzyme solution (60 mL) were incubated for 5 min at 25°C. Likewise, AA (30 mM; 20 mL) was added to initiate the reaction and allowed to stand for 4–5 min. Afterwards, the absorbance (Abs) of the control and test samples was noticed at 570 nm through a ultraviolet–visible (UV–vis) spectrophotometer. The COX‐2 enzyme's percent inhibition was calculated using the absorbance value per unit of time. The IC_50_ values were calculated by creating a graph comparing the inhibition and concentration of the tested sample solution. In this assay, Celecoxib was used as a reference drug.

#### 2.5.2 5‐LOX assay

The 5‐LOX assay was also performed to evaluate the anti‐inflammatory potential of *A. nilotica*'s crude methanolic extract by following the methods of Jan et al. (2019). Purposely, different concentrations of the extract (62.5–1000 mg mL^−1^) were made in this assay. Subsequently, a 5‐LOX enzyme solution comprising 10,000 U mL^−1^ of 5‐LOX enzyme was prepared. Linoleic acid (80 mM) was used as a substrate to start the reaction. Moreover, a phosphate buffer (250 mL; 50 mM; pH 6.3) was mixed with crude extracts, followed by adding enzyme solution (250 mL) and incubating for 5 min. After that, a substrate solution (500 mL) was mixed with an enzyme solution with continuous agitation. The absorbance (Abs) of control and test samples was examined at 234 nm via a ultraviolet–visible (UV–vis) spectrophotometer. Montelukast was used as a positive control in this assay. In the end, the percent inhibition of 5‐LOX was calculated using the following formula:

$$\%\text{inhibition}=\left[\frac{\mathrm{Abs}.\;\text{of control}-\mathrm{Abs}.\;\text{of test sample}}{\mathrm{Abs}.\;\text{of control}}\right]\times 100$$

RETRACTED

### 2.6 Statistical analysis

Results in this study were presented as mean ± SEM. Student's *t* test was performed to compare the inhibitory effects of standard drugs and *A. nilotica*'s methanolic extracts. *p*‐Value <.05 values was considered significant.

## 3 RESULTS

### 3.1 Antidiabetic effect

The α‐glucosidase and α‐amylase activities of the crude methanolic extract of *Acacia nilotica* are summarized in Table 1. All the tested concentrations (62.5–1000 μg mL^−1^) of crude extract and standard drug (acarbose) showed percent inhibition of α‐glucosidase in the range of 58.74%–77.34% and 59.12%–81.85%, respectively. Similarly, the α‐amylase percent inhibition of the extract was noticed as 62.98%, 67.90%, 72.91%, 77.08%, and 81.03% with an IC_50_ value of 17.00 μg mL^−1^ at the concentrations 62.5, 125, 250, 500, and 1000, respectively. On the other hand, the percent inhibition of α‐amylase of the standard drug (62.5–1000 μg mL^−1^) was reported as 61.35, 66.20, 73.42, 78.62, and 83.53, respectively, with IC_50_: 21.30 μg mL^−1^. At maximum concentration (1000 μg mL^−1^), the α‐glucosidase inhibitory activity of extract was lower (77.34%), as compared to that of standard drug (81.85%). While, the α‐amylase percent inhibitory activity of extract at maximum concentration (1000 μg mL^−1^) was comparable (81.03%) to that of standard drug (83.53%).

**TABLE 1:** Antidiabetic activity of methanolic extract of *Acacia nilotica*.

Samples	Concentration (μg mL^−1^)	% α‐glucosidase (mean ± SEM)	IC_50_ (μg mL^−1^)	% α‐amylase (mean ± SEM)	IC_50_ (μg mL^−1^)
*Acacia nilotica*	1000	77.34 ± 0.98^ns^	33	81.03 ± 0.35^ns^	17
	500	72.32 ± 1.06^ns^		77.08 ± 0.47^ns^	
	250	67.05 ± 0.75^ns^		72.91 ± 0.88^ns^	
	125	62.70 ± 1.25^ns^		67.90 ± 0.96^ns^	
	62.5	58.74 ± 0.68^ns^		62.98 ± 0.72^ns^	
Acarbose	1000	81.85 ± 0.18	26.58	83.53 ± 0.20	21.30
	500	76.59 ± 0.30		78.62 ± 0.17	
	250	69.75 ± 0.14		73.42 ± 0.11	
	125	64.47 ± 0.49		66.20 ± 0.15	
	62.5	59.12 ± 0.34		61.35 ± 0.18	

*Note*: The effect of tested crude extract on antidiabetic activity. The values are expressed as mean ± SEM. ns (non‐significant) compared to standard drugs (Acarbose). Data were analyzed via Student's *t* test.

RETRACTED

### 3.2 Anticholinesterase effect

Results of this assay revealed that the crude methanolic extract of *A. nilotica*, when administered at different concentrations (62.5–1000 μg mL^−1^), displayed substantial (*p* < .05) cholinesterase‐inhibiting effects, as demonstrated in Table 2. The results showed that the AChE percent inhibition was 67.54%, 35.02%, 29.69%, 21.72%, and 15.35% at concentrations ranging from 1000, 500, 250, 125, and 62.5 μg mL^−1^, respectively, with an IC_50_ value of 637.01 μg mL^−1^. The standard drug Galantamine exhibited 82.43%, 74.03%, 71.56%, 67.05%, and 63.26% AChE percent inhibition with an IC_50_ value of 12.63 μg mL^−1^. Likewise, the BChE percent inhibition was measured as 71.50, 41.61, 34.22, 24.90, and 17.36 at concentrations ranging from 1000, 500, 250, 125, and 62.5 μg mL^−1^, respectively, with an IC_50_ value of 491.98 μg mL^−1^. Similarly, the standard drug (Galantamine) displayed 89.50, 83.00, 77.50, 73.53, and 67.63 BChE percent inhibition, causing an IC_50_ value of 10.57 μg mL^−1^ (Table 2). At maximum concentration (1000 μg mL^−1^), the AChE inhibitory activity of the extract was significantly lower (67.54%) as compared to that of the standard drug (82.43%). Similarly, the BChE percent inhibitory activity of the extract at maximum concentration (1000 μg mL^−1^) was also significantly lower (71.50%) than that of the standard drug (89.50%).

**TABLE 2:** Anticholinesterase activity of methanolic extract of *Acacia nilotica*.

Samples	Concentration (μg mL^−1^)	% AChE (mean ± SEM)	IC_50_ (μg mL^−1^)	% BChE (mean ± SEM)	IC_50_ (μg mL^−1^)
*Acacia nilotica*	1000	67.54 ± 0.38***	637.01	71.50 ± 0.27***	491.98
	500	35.02 ± 0.21***		41.61 ± 0.24***	
	250	29.69 ± 0.63***		34.22 ± 0.06***	
	125	21.72 ± 0.34***		24.90 ± 0.23***	
	62.5	15.35 ± 0.19***		17.36 ± 0.43***	
Galantamine	1000	82.43 ± 0.52	12.63	89.50 ± 1.00	10.57
	500	74.03 ± 0.64		83.00 ± 0.00	
	250	71.56 ± 0.49		77.50 ± 0.57	
	125	67.05 ± 0.49		73.53 ± 0.55	
	62.5	63.26 ± 0.93		67.63 ± 0.33	

*Note*: The effect of tested crude extract on anticholinesterase activity. The values are expressed as mean ± SEM. ***p < .001 compared to standard drugs (Galantamine). Data were analyzed via student *t* test.

### 3.3 In vitro anti‐inflammatory analysis

#### 3.3.1 Cyclooxygenase 2 (COX‐2) inhibitory effect

The dose‐dependent activity of the *A. nilotica* in Table 3 showed substantial reductions in COX‐2 activity. The crude extract of *A. nilotica* exhibited 75.22%, 79.62%, 61.75%, 57.53%, and 43.48% inhibition (IC_50_: 83.03 μg mL^−1^) at concentrations 1000, 500, 250, 125, and 62.5 μg mL^−1^, respectively. Moreover, the standard drug (Celecoxib) exhibited 95.20%, 91.17%, 86.98%, 81.20%, and 77.80% inhibition (IC_50_ 3.22 μg mL^−1^) at concentrations 1000, 500, 250, 125, and 62.5 μg mL^−1^ respectively. Results revealed that as compared to standard drug (Celecoxib; 95.20%), the percent COX‐2 inhibitory activity of the extract was significantly lower (75.22%) at maximum concentration (1000 μg mL^−1^).

RETRACTED

**TABLE 3:** Percent COX‐2 and 5‐LOX inhibition activity of methanolic extract of *Acacia nilotica*.

Samples	Concentration (μg mL^−1^)	% COX‐2 inhibition	IC_50_ (μg mL^−1^)	% 5‐LOX inhibition	IC_50_ (μg mL^−1^)
*Acacia nilotica*	1000	75.22 ± 0.47***	83.03	71.53 ± 0.49***	76.82
	500	79.62 ± 0.36***		68.46 ± 0.63***	
	250	61.75 ± 0.58***		63.31 ± 0.57***	
	125	57.53 ± 0.71***		60.34 ± 0.65***	
	62.5	43.48 ± 0.50***		42.47 ± 0.55***	
Celecoxib	1000	95.20 ± 0.15	3.22	—	—
	500	91.17 ± 0.53		—	
	250	86.98 ± 0.85		—	
	125	81.20 ± 0.65		—	
	62.5	77.80 ± 0.37		—	
Montelukast	1000	—	—	93.55 ± 0.40	4.50
	500	—		89.37 ± 1.65	
	250	—		85.50 ± 0.40	
	125	—		79.60 ± 0.90	
	62.5	—		74.17 ± 0.72	

*Note*: The effect of tested crude extract on anti‐inflammatory activity. The values are expressed as mean ± SEM. ***p < .001 compared to standard drugs (Celecoxib for COX‐2 and Montelukast for 5‐LOX). Data were analyzed via Student's *t* test.

#### 3.3.2 5‐LOX inhibitory effect

The studied *A. nilotica* crude methanolic extract was evaluated for 5‐LOX inhibitory potential. The anti‐5‐LOX activity of the *A. nilotica* extract is shown in Table 3. The extract displayed 5‐LOX inhibition (IC50: 76.82 μg mL^−1^) in the range of 42.47–71.53% at varied (62.5–1000 μg mL^−1^) concentrations. The standard drug (Montelukast) inhibited 5‐LOX activity with an IC_50_ value of 4.50 μg mL^−1^ (Table 3). The 5‐LOX percent inhibitory activity of the extract at maximum concentration (1000 μg mL^−1^) was observed to be significantly lower (71.53%) than that of the standard drug (Montelukast; 93.55%).

## 4 DISCUSSION

Natural compounds in plant extracts have shown hypoglycemic properties, besides their antioxidant capabilities by binding to glucose transporters and inhibiting digestive enzymatic activity (Baldea et al., 2010; Lacroix & Li‐Chan, 2014). α‐Amylase and α‐glucosidase are the most critical hydrolyzing enzymes that break down starch from food and convert oligosaccharides into glucose, leading to a spike in blood sugar levels after a meal. Therefore, inhibiting their functionality is crucial for managing hyperglycemia in type 2 DM patients. The current study revealed a significant inhibitory effect of crude methanolic extract of *A. nilotica* against α‐amylase and α‐glucosidase (Table 1). The results of our study are in accordance with the previous research conducted by Elbashir et al. (2018). They reported that an extract of *A. nilotica* found in Sudan demonstrated significant in vitro antidiabetic activity by inhibiting α‐glucosidase activity. Earlier, Vadivel and Biesalski (2012) also showed a similar inhibitory (72.91%) potential of *A. nilotica*'s seed extract against α‐amylase.

RETRACTED

The widespread prevalence and associated high mortality of neurological disorders have made them a primary global health concern. Currently, in clinical practice, few drugs help effectively treat neurological problems without causing harmful side effects. Natural components are a promising solution due to their significant bioactivities and accessibility to humans. Thus, they are considered an essential alternative for developing novel drugs to treat neurological disorders (Anand et al., 2017). Elevated activity of the AChE and BChE reduces vital neurotransmitters, i.e., ACh and butyrylcholine (BCh) levels. Hence, AChE and BChE inhibitory agents are considered viable options for elevating the levels of ACh and BCh, respectively (Long & Holtzman, 2019; Pardridge, 2020; Sonawane et al., 2021; Vaz & Silvestre, 2020). In this study, crude methanolic extract of *A. nilotica* significantly inhibited the activity of AChE (67.54%) and BChE (71.50%), as compared to the standard drug (82.43 and 89.50%, respectively). The cholinesterase inhibitory activity of crude extract indicates the therapeutic potential of *A. nilotica* against neurological disorders. According to a study, an aqueous extract of *A. nilotica* roots possesses AChE inhibitory activity (Eldeen et al., 2010). Similarly, Niloticane, a bioactive component of *A. nilotica*, has also shown antiacetylcholinesterase activity with a reported IC_50_ value of 4 μM (Osama et al., 2015). Another group of researchers revealed the AChE inhibitory potential (0.35–5.40 μg mL^−1^) of extracts (ethyl acetate, butanol, aqueous, and chloroform) of *A. nilotica* pods (Crowch & Okello, 2009).

The COX and LOX pathways are vital in causing inflammation and related pain (American Diabetes Association, 2010). Inhibitors of these pathways interrupt the production of prostaglandins and leukotrienes, which are responsible for inflammation (Leval et al., 2002). Hence, halting these pathways by inhibiting COX‐2 and 5‐LOX enzymes effectively reduces inflammation. Selective COX‐2 inhibition is beneficial in developing anti‐inflammatory drugs (Mendes et al., 2012). The LOX enzyme family, which contains iron, catalyzes AA's oxygenation, and each LOX generates a distinct 5‐hydroperoxyeicosatetraenoic acid (5‐HPETE) (Mahnashi et al., 2021). Four types of LOX exist, such as 5‐LOX, 8‐lipoxygenase (8‐LOX), 12‐lipoxygenase (12‐LOX), and 15‐lipoxygenase (15‐LOX), which are found in animals, plants, and fungi (Khan et al., 2021). The 5‐LOX protein is mainly present in myeloid cells, lymphocytes, macrophages, and monocytes, vital in inflammatory and immune responses. Stimuli that activate 5‐LOX and initiate leukotriene synthesis include interleukin 8 (IL‐8), Ca^+2^ mobilizing agents, phagocytic particulates, and the complement peptide C5a (Munir et al., 2020). During the in vitro 5‐LOX and COX‐2 inhibitory assay conducted in this study, we noticed that varied concentrations (62.5–1000 μg mL^−1^) of crude methanolic extract of *A. nilotica* selectively inhibited 5‐LOX (42.47%–71.53%) and COX‐2 (43.48%–79.62%) activities with IC_50_ values of 76.82 μg mL^−1^ and 83.03 μg mL^−1^, respectively. The results depicted in our study were in accordance with earlier reported data (Magaji, 2022; Niyodusenga et al., 2019; Srivastava & Mishra, 2020). Results of the present study revealed in vitro antidiabetic, anti‐inflammatory, and anti‐AChE activity of crude methanolic extract of *A. nilotica*. However, further experimental investigations are needed to validate these potentialities.

RETRACTED

## 5 CONCLUSIONS

It can be concluded from the results of our current research that *A. nilotica* possesses varied bioactivities. Herein, we evaluated the in vitro antidiabetic property of *A. nilotica*'s crude methanolic extract. We confirmed that *A. nilotica* inhibited the activity of α‐amylase and α‐glucosidase with IC_50_ values of 17 and 33 μg mL^−1^, respectively. COX‐2 and 5‐LOX activities were also inhibited (43.48%–79.62% and 42.47%–71.53%) by varied concentrations of *A. nilotica* extract. Moreover, the experimented extract significantly inhibited the activity of cholinesterase (AChE and BChE). In a nutshell, these results will provide the scientific community with baseline data in planning and executing further in vivo and clinical studies to investigate the use of *A. nilotica* to treat or support treatment diabetes, inflammation, and AD.

## AUTHOR CONTRIBUTIONS

**Abdur Rauf:** Conceptualization (equal); data curation (equal); formal analysis (equal); methodology (equal); project administration (equal); supervision (equal); writing – original draft (equal); writing – review and editing (equal). **Muhammad Ibrahim:** Conceptualization (equal); data curation (equal); formal analysis (equal); methodology (equal); writing – review and editing (equal). **Taghrid S. Alomar:** Data curation (equal); investigation (equal); methodology (equal); resources (equal); writing – original draft (equal). **Najla AlMasoud:** Data curation (equal); investigation (equal); methodology (equal); validation (equal); visualization (equal). **Anees Ahmed Khalil:** Conceptualization (equal); data curation (equal); investigation (equal); supervision (supporting); writing – original draft (equal); writing – review and editing (equal). **Muneeb Khan:** Data curation (equal); methodology (equal); visualization (equal); writing – original draft (equal); writing – review and editing (equal). **Ahood Khalid:** Formal analysis (equal); methodology (equal); visualization (equal); writing – original draft (equal); writing – review and editing (equal). **Muhammad Saeed Jan:** Conceptualization (supporting); data curation (supporting); investigation (equal); project administration (equal); validation (equal); writing – original draft (equal). **Dorota Formanowicz:** Conceptualization (equal); funding acquisition (equal); methodology (equal); resources (equal); visualization (equal); writing – original draft (equal); writing – review and editing (equal). **Mohammed Mansour Quradha:** Conceptualization (equal); methodology (equal); project administration (equal); software (equal); writing – original draft (equal); writing – review and editing (equal).

RETRACTED

## CONFLICT OF INTEREST STATEMENT

The authors declare that they have no known competing financial interests or personal relationships that could have appeared to influence the work reported in this paper.

## Data Availability

The data associated with this paper are given in the main text of this manuscript.
